# Characterization of the Modulatory Effect of Hydroxychloroquine on ACE2 Activity: New Insights in relation to COVID-19

**DOI:** 10.1155/2021/6614000

**Published:** 2021-07-23

**Authors:** Juan E. Tichauer, Dagoberto Soto, Max Andresen

**Affiliations:** Department of Intensive Care Medicine, School of Medicine, Pontificia Universidad Católica de Chile, Santiago/8330024, Chile

## Abstract

Chloroquine (CQ) and hydroxychloroquine (HCQ) have shown the ability to inhibit *in vitro* viral replications of coronaviridae viruses such as SARS-CoV and SARS-CoV-2. However, clinical trial outcomes have been disparate, suggesting that CQ and HCQ antiviral mechanisms are not fully understood. Based on three-dimensional structural similarities between HCQ and the known ACE2 specific inhibitor MLN-4760, we compared their modulation on ACE2 activity. Here we describe, for the first time, in a cell-free *in vitro* system that HCQ directly and dose-dependently inhibits the activity of recombinant human ACE2, with a potency similar to the MLN-4760. Further analysis suggests that HCQ binds to a noncompetitive site other than the one occupied by MLN-4760. We also determined that the viral spike glycoprotein segment that comprises the RBD segment has no effect on ACE2 activity but unexpectedly was able to partially reverse the inhibition induced by HCQ but not that by MLN-4760. In summary, here we demonstrate the direct inhibitory action of HCQ over the activity of the enzyme ACE2. Then, by determining the activity of ACE2, we reveal that the interaction with the spike protein of SARS-CoV-2 leads to structural changes that at least partially displace the interaction of the said enzyme with HCQ. These results may help to explain why the effectiveness of HCQ in clinical trials has been so variable. Additionally, this knowledge could be used for to develop techniques for the detection of SARS-CoV-2.

## 1. Introduction

Chloroquine (CQ) and its less toxic derivative hydroxychloroquine (HCQ) have shown *in vitro* to efficiently inhibit viral replication, including strains of coronaviridae virus SARS-CoV [1–4] and SARS-CoV-2 [5]. As coronaviridae viruses infect their target cells through an endocytic pathway [6, 7], it has been proposed that the mechanism of action of CQ and HCQ is mediated by the acidification of organelles such as the endosome, Golgi vesicles, and the lysosomes. CQ and HCQ prevent the attachment of the virus by interfering with sialic acid biosynthesis, which is critical in virus-cell recognition. Furthermore, once the virus is internalized, CQ and HCQ hinder the vesicle maturation and releasing of viral genome, preventing the replication and spread of the virus [8–10]. The use of HCQ as a treatment for SARS-CoV-2 has been proposed, mainly based on its effectiveness demonstrated *in vitro*. In fact, nowadays, there are more than 200 clinical trials evaluating its therapeutic value (https://clinicaltrials.gov/ct2/home). Until now, the results of these trials have been variable, ranging from an encouraging decrease in nasopharyngeal viral load to some indifferent and even harmful clinical outcomes. This variety of results strongly suggests that the mechanics behind the antiviral action of HCQ is still not fully known. Thus, the HCQ antiviral mechanism is still awaiting to be revealed.

The first step in host infection by SARS-CoV-2 is the recognition and interaction of the RBD segment at viral spike glycoprotein with the angiotensin-converting enzyme 2 (ACE2) [11, 12]. One could believe that this interaction modulates the activity of ACE2 and in turn be useful as a diagnostic tool, or alternatively, that the modulation of the activity could conveniently modulate the infection by SARS-CoV-2. However, it was shown that the presence of the spike glycoprotein does not exert modulating on the proteolytic activity of ACE2 on its substrates. Moreover, the highly selective inhibitor MLN-7460 does not limit the viral infection by SARS-CoV-2 [13]. The preceding data discouraged further investigations linking ACE2 and SARS-CoV-2 activity. In this work, we demonstrate that in a cell-free *in vitro* system, HCQ directly and dose-dependently inhibits the activity of recombinant human ACE2. The presence of the viral spike glycoprotein segment comprising the RBD segment reversed the inhibition induced by HCQ but not that by MLN-4760. Those results reveal new pharmaceutical targets of HCQ and suggest the development of potential new diagnostic procedures to determine the presence of SARS-CoV-2.

## 2. Material and Methods

Recombinant Human ACE2 protein and Recombinant Human Coronavirus SARS-CoV-2 Spike Glycoprotein RBD (Active) (ab151852 and ab273065, respectively) were purchased from ABCAM; MLN-4760 (Cat. No.: HY-19414-10) was purchased from https://www.medchemexpress.com/, and SensoLyte®390 ACE2 Activity Assay Kit (AS-72086) was purchased from https://www.anaspec.com; HCQ was purchased from a local pharmaceutical provider.

The ACE2 activity was measured in a Microplate Spectrophotometer Synergy™ 2 (Biotek, USA) using the SensoLyte®390 kit in a kinetic mode (10 seconds steps) during the whole time. The experimental optimization showed that in the absence of enzyme, the substrate (Mc-Ala/Dnp) does not show a measurable change in its level of fluorescence over time. Kinetics were evaluated in multiple concentrations of rhACE2 (5-500 ng/ml); 5 ng/ml was chosen because it exhibited a good signal-to-noise ratio, as it exhibited a linear product synthesis rate range of at least 1.5 hours. HCQ was prepared the same day of assays from a 100 *μ*M stock to a final concentration in the well. HCQ has an interfering emission at 390 nm that was evaluated and determined as constant and that does not show interaction with MCA or DNP, so that the baseline of said experiments was contrasted with the emission kinetics observed in a reaction medium comprising the same reaction components in the absence of the rhACE2 enzyme. Spike glycoprotein RBD was used from a 200 *μ*g/ml stock and diluted to a final concentration of 100 nM in the well. The percentage of loss of rhACE2 activity induced by the different modulators was calculated with respect to the control situation in the absence of inhibitor.

## 3. Statistical Analysis

Results were analyzed using a Mann–Whitney nonparametric test using the GraphPad Prism v.5.0 (GraphPad Software). *P* values < 0.05 were considered to indicate statistical significance.

## 4. Results

### 4.1. HCQ Inhibits rhACE2

The three-dimensional structures of the HCQ (PubChem CID; 3652) and the MLN-4760 (PubChem CID; 448281) display a relatively similar structural domain. Both molecules comprise a halogen substituted aromatic ring and in a “para” location exhibit a 6-8 atom radical substitution ending in one or more alcoholic or carboxylic groups. These similarities motivated us to evaluate a possible similar modulation on the ACE2 enzyme. Indeed, HCQ inhibited directly and dose-dependently the activity of rhACE2 (5 ng/ml), with a comparable efficiency (-log Ki = 7.49) to the known selective inhibitor MLN-4760 (-log Ki = 7.86) (Figure 1).

### 4.2. Modulation of ACE2 Activity by SARS-CoV-2 Spike Glycoprotein and Its Interaction with Inhibitors MLN-4760 and HCQ

Recently, Nami et al. using computational modeling predicted that the binding SARS-CoV-2 spike RBD to ACE2 (MLN-4760) abrogates the inhibitory effect of MLN-4760. We tested this hypothesis using both MLN-4760 and HCQ as inhibitors. In each case, we use concentrations of these compounds close to their –log Ki in order to set a similar dynamic range allowing us to detect a potential “loss-inhibition” of the preinhibited ACE2 (Figures 1 and 2(a)). Consistent with the previous literature, we found that spike glycoprotein by itself did not have any effect on ACE2 activity under the measured condition (Figures 2(b) and 2(c)). Contrary to what was predicted, the presence of spike glycoprotein had no effect on ACE2 preinhibited with 50 nM MLN-4760 (58.4 ± 7.4 vs. 53.5 ± 11.4% of ACE2 activity in the absence or presence of spike glycoprotein) (Figures 2(b) and 2(d)). Surprisingly, spike glycoprotein was able to partially restore the activity of the enzyme preinhibited with the molecule 100 nM HCQ (67.06 ± 8.1 vs. 86 ± 7.1% of ACE2 in the absence or presence of spike glycoprotein) (Figures 2(b) and 2(e)). Furthermore, we found that the combined effect of MLN-4760 and HCQ in the range of their Ki led to an inhibition which was the arithmetic sum of the independent inhibitions (Figures 2(a) and 2(f)).

## 5. Discussion

Motivated by putative structural analogies, in this cell-free model, we demonstrated that HCQ directly and dose-dependently inhibited ACE2 activity. Interestingly, when HCQ and MLN-4760 were coincubated, there was an additive inhibition. The latter suggests that the sites of action of these agents would not be the same.

Nami et al. and Teralı et al. described *in silico* models where the binding of ACE2 to the selective inhibitor MLN-4760 predicts conformational changes, which modify the enzymatic active site and alter the binding site and residues involved in the hydrogen and hydrophobic binding between spike glycoprotein RBD domain and ACE2 [13, 14]. Nami et al. also put forward that spike glycoprotein can rescue the enzymatic activity of the MLN-4760 inhibited ACE2. In opposition to that hypothesis in our *in vitro* system, spike glycoprotein was not able to reestablish the activity of the MLN-4760 inhibited ACE2 enzyme. Unexpectedly, spike glycoprotein partially restored the activity of ACE2 preinhibited with HCQ, indicating, for the first time, that the SARS-CoV-2/host structural interaction is NOT ACE2 activity-independent. This new antecedent and its possible implications, both in the cellular context of signal transduction and in the physiological context due to the forced ACE2 activity, must be considered for a future explanation of the until now inability to transfer the antiviral effect of HCQ to the clinic.

Considering that (a) we have detected the presence of ACE2 in saliva through the methodology used in this study (data no shown) and (b) the presence of the virus in saliva is known in subjects who are positive for COVID-19 [15], we believe that the changes demostrated in the ACE2 activity preinhibited by HCQ induced by the spike glycoprotein of SARS-CoV-2 could be conveniently used as a diagnostic tool to evaluate the presence of the said virus in saliva.

## Figures and Tables

**Figure 1:** Inhibition of ACE2 activity by different concentrations on MLN-4760 or HCQ. Graph shows % of inhibition for ACE2 activity in an inhibitory activity *in vitro* assay using different concentrations of the specific ACE2 blocker MLN-4760 (black circles) and the aminoquinoline HCQ (diamonds). *n* = 3‐5.

**Figure 2:** Modulation of ACE2 activity by SARS-CoV-2 spike glycoprotein and its interaction with the inhibitors MLN-4760 and HCQ. Enzyme activity was assayed in the presence of SARS-CoV-2 spike protein (SP), ACE2 inhibitor MLN4760 (MLN), aminoquinoline hydroxychloroquine (HCQ), or their combinations. (a) ACE2 activity in presence of HCQ, MLN4760, or its combination was measured in a kinetic assay using the SensoLyte®390 kit. Fluorescence level and linear regression are represented for each reaction. (b) Kinetic assay showing the effect of SP on HCQ inhibition. (c) Quantification of the effect of SP, MLN, and HCQ on ACE2 activity. SP effect on the inhibition of ACE2 produced by (d) MLN and (e) HCQ. (f) Combined effect HCQ and MLN on ACE2 activity. Relevant comparisons are shown within brackets. ^∗^*P* < 0.05. *n* = 3‐5.

## Data Availability

The datasets used and/or analyzed during the current study are available from the corresponding author on reasonable request.

## Abbreviations

ACE2: Angiotensin-converting enzyme 2
HCQ: Hydroxychloroquine
SP: Spike glycoprotein.
